# Identification of Molecular Targets and Underlying Mechanisms of Xiaoji Recipe against Pancreatic Cancer Based on Network Pharmacology

This article has been retracted.

**DOI:** 10.1155/2022/4640849

**Published:** 2022-09-08

**Authors:** Cunbing Xia, Dexuan Chen, Gaoyuan Wang, Haijian Sun, Jingran Lin, Chen Chen, Tong Shen, Hui Cheng, Chao Pan, Dong Xu, Hongbao Yang, Yongkang Zhu, Hong Zhu

**Affiliations:** ^1^Department of General Surgery, Affiliated Hospital of Nanjing University of Chinese Medicine, Jiangsu Province Hospital of Chinese Medicine, Nanjing, Jiangsu 210029, China; ^2^The Inheriting Studio of National Famous Old Chinese Medicine Experts-Zhu Yongkang (National Traditional Chinese Medicine Science and Education 2022 No. 75), Nanjing, Jiangsu 210029, China; ^3^Pancreas Center, The First Affiliated Hospital of Nanjing Medical University, Nanjing, Jiangsu 210029, China; ^4^Center for New Drug Safety Evaluation and Research, Institute of Pharmaceutical Science, China Pharmaceutical University, Nanjing, Jiangsu 211198, China

## Abstract

Traditional Chinese medicine (TCM) is applied in the anticancer adjuvant therapy of various malignancies and pancreatic cancer included. Xiaoji recipe consists several TCM materials with anticancer activities. In our work, we intended to analyze the molecular targets as well as the underlying mechanisms of Xiaoji recipe against pancreatic cancer. A total of 32 active components and 522 potential targets of Xiaoji recipe were selected using the TCMSP and SwissTargetPrediction databases. The potential target gene prediction in pancreatic cancer was performed using OMIM, Disgenet, and Genecards databases, and totally, 998 target genes were obtained. The component-disease network was constructed using the Cytoscape software, and 116 shared targets of pancreatic cancer and Xiaoji recipe were screened out. As shown in the protein–protein interaction (PPI) network, the top 20 hub genes such as TP53, HRAS, AKT1, VEGFA, STAT3, EGFR, and SRC were further selected by degree. GO and KEGG functional enrichment analysis revealed that Xiaoji recipe may affect pancreatic cancer progression by targeting the PI3K/AKT and MAPK signaling pathways. Moreover, we performed *in vitro* assays to explore the effect of Xiaoji recipe on pancreatic cancer cells. The results revealed that Xiaoji recipe suppressed the viability and migration and promoted the apoptosis of pancreatic cancer cells via the inactivation of PI3K/AKT, MAPK, and STAT3 pathways. The findings of our study suggested the potential of Xiaoji recipe in the targeting therapy of pancreatic cancer.

## 1. Introduction

Pancreatic cancer is a fatal malignancy and ranks the seventh leading cause of cancer-related death in both sexes, with approximately 5 million new cases and 466000 death cases in 2020 [1]. Many risk factors may contribute to the development of pancreatic cancer, including genetic background, obesity, type II diabetes, and tobacco smoking [2]. The chemotherapy with gemcitabine is regarded as the first-line treatment for pancreatic cancer, with 23.8% clinical response and a 5-year survival rate of 2% [3, 4]. However, the prognosis of pancreatic cancer patients is still unsatisfactory due to the late diagnosis, early metastasis, and limited chemotherapy effects [5]. Therefore, it is imperative to investigate potent treatment options to improve the clinical outcome of anticancer therapy in pancreatic cancer.

Traditional Chinese medicine (TCM), especially Chinese herbal medicines and acupuncture, is used to treat advanced cancers with low-toxic effects and is reported to increase physical function, reduce symptoms, and improve the life quality of patients [6, 7]. Increasing studies have demonstrated the antitumor effects of TCM on the proliferation, metastasis, and tumorigeneis in cancer development [8]. In pancreatic cancer, it has been reported that scoparone inhibits tumor progression via PI3K/Akt signaling pathway [9]. Besides, a proteoglycan extracted from *Ganoderma lucidum* can induce cancer cell apoptosis [10]. The prescription of Xiaoji recipe is mainly composed of *Curcuma zedoaria* (10 g, E Zhu), *Polygonum cuspidatum* (10 g, Huzhang), *clematis root* (10 g, Weilingxian), *Rhizoma Paridis* (10 g, Zhonglou), and *Eupolyphaga Steleophaga* (10 g, Tubiechong). The main functions of Xiaoji recipe is to eliminate the heat and dampness and promote the blood circulation and can be used in the antitumor therapy for various cancers. *Curcuma zedoaria* (Zingiberaceae) is reported to inhibit the development of gastric carcinoma, breast cancer as well as liver cancer [11–14]. *Polygonum cuspidatum* is used for the therapy of multiple diseases including hypertension, diabetes, and atherosclerosis [15–17], and its extracts have been reported with anticancer effects in lung cancer, osteosarcoma, and breast cancer [18–20]. The extracts of *Rhizoma Paridis* is revealed to suppress the cancer development in non-small-cell lung carcinoma, colon cancer, and hepatocarcinoma [21–23]. *Eupolyphaga Steleophaga* is reported to be used in the treatment of fractures, falls, uterine fibroids, or menstrual problems [24], while its effects in cancer are not fully understood.

Network-based pharmacology is widely used in drug discovery by predicting potential mechanisms via exploring the targets of drugs, diseases, and their biomolecular networks [25, 26]. In TCM, a holistic perspective has long been at the heart of the herbal treatment of various diseases. TCM prescriptions have holistic theory and rich experience in multicomponent therapy, which provides a bright prospect for systematic treatment of complex diseases. Therefore, linking emerging network science with ancient TCM will provide new methods and opportunities to discover bioactive components and biomarkers, reveal mechanisms of action, and explore the scientific basis of TCM formulations based on complex biological systems [27]. Moreover, network-based pharmacology is becoming a frontier research field in current cancer drug research. For example, Huang et al. have explored the potential effect of Tao Hong Si Wu decoction for treating breast cancer according to network pharmacology and experimental [28].

Signaling pathways such as the phosphoinositide 3 kinase/AKT (PI3K/AKT) signaling pathway, signal transducer and activator of transcription 3 (STAT3) signaling pathway, and mitogen-activated protein kinases (MAPK) signaling pathway are important in the pathological process of pancreatic cancer and are frequently activated in pancreatic cancer. They are associated with poor prognosis of pancreatic cancer. Aberrant activation of these pathways are involved in cell survival, cell cycle progression, and cell apoptosis [29, 30]. Targeting these signaling pathways may be an approach to cancer treatment.

In our study, we intended to explore the potential core targets and pathways of Xiaoji recipe against pancreatic cancer based on the TCM network pharmacology approach. The findings of our study may provide clues for the targeting therapy of Xiaoji recipe in pancreatic cancer.

## 2. Materials and Methods

### 2.1. Cell Culture and Treatment

Pancreatic cell lines (CFPAC (cat. no. CRL-1918; PANC1, cat. no. CRL-1469)) were provided by the ATCC (American Type Culture Collection, USA), CFPAC cell line was cultured in Iscove's modified Dulbecco's medium. PANC1 cell line was cultured in Dulbecco's modified Eagle's medium (DMEM, Cytiva, Shanghai, China). Both culture mediums were maintained in an incubator supplemented with g 10% FBS (Beyotime, Shanghai, China) at 37°C and 5% CO_2_. To evaluate the effects of Xiaoji recipe on cell malignant behaviors *in vitro*, the CFPAC and PANC1 cells were treated with 150 *μ*g/ml or 300 *μ*g/ml Xiaoji recipe.

### 2.2. Cell Viability

The viability of pancreatic cancer cells was measured using a Cell Counting Kit-8 (CCK-8; MCE, Inc., Shanghai, China). The treated CFPAC and PANC1 cells were grown into 96-well plates at 2000 cells/well and incubated for 24, 48, and 72 h, followed with addition of 10 *μ*l CCK-8 solution, followed with incubation for another 2 h at 37°C. A microplate reader (HBS-1096A, DeTie Laboratory Equipment Co., Ltd., Nanjing, China) was used to determine the absorbance at 450 nm.

### 2.3. Wound Healing Assay

The treated CFPAC and PANC1 cells were plated into 6-well plates supplemented with medium and 1.5% fetal bovine serum and cultured to reach 90% confluence. Then, the plates were scratched using a 10 *μ*l pipette tip. A microscope (Olympus, Shanghai, China) was used to photograph the wound healing distance at 0 and 48 h.

### 2.4. Flow Cytometry Analysis

The apoptosis of CFPAC and PANC1 cells after indicated treatments was assessed by flow cytometry analysis. CFPAC and PANC1 cells were harvested, washed with PBS, and resuspended in a 500 *μ*l mixture with 5 *μ*l Annexin and 10 *μ*l propidium iodide (7-AAD; MultiSciences Biotech, Co., Ltd., Hangzhou, China). Finally, cell apoptosis rate was detected using a flow cytometer and analyzed with the FlowJo software. The apoptosis rate in each group was calculated by Q2 (late apoptosis) + Q3 (early apoptosis).

### 2.5. Western Blot

RIPA lysis buffer (Beyotime, Shanghai, China) was used to collect the protein in treated CFPAC and PANC1 cells. The concentration of collected proteins was evaluated using a BCA Protein Assay kit (Beyotime, Shanghai, China). Then, the proteins were separated with 10% SDS-PAGE gels and electrotransferred on the PVDF membranes. The Protein-Free Rapid Blocking Buffer (Epizyme, Shanghai, China) was used to block the membranes for 1 h, which were then cultured with the primary antibodies against AKT1 (1 : 1000, Abcam, USA), STAT3 (1 : 1000, Abcam, USA), EGFR (1 : 1000, Abcam, USA), MAPK3 (1 : 1000, Abcam, USA) at 4°C overnight, and GAPDH (1 : 1000, Abcam, USA) served as an internal reference. Next, the membranes were washed with TBST and cultured with corresponding secondary antibodies (1 : 2000, Abcam, USA) for 2 h at room temperature. Finally, the protein signal was detected using a Biosharp ECL detection kit (Biosharp, Beijing, China) and analyzed with ImageJ software.

### 2.6. Exploration of Active Components and Potential Targets of Xiaoji Recipe

Xiaoji recipe is a traditional Chinese prescription composed of *Curcuma zedoaria* (E Zhu), *Polygonum cuspidatum* (Huzhang), *clematis root* (Weilingxian), *Rhizoma Paridis* (Zhonglou), and *Eupolyphaga Steleophaga* (Tubiechong). The active components of these TCM materials were searched on the Traditional Chinese Medicine Systems Pharmacology Database and Analysis Platform (TCMSP, http://lsp.nwu.edu.cn/tcmsp.php) [31] under the condition of oral bioavailability (OB) ≥ 30% and drug − likeness (DL) ≥ 0.18 and TCMID database (http://119.3.41.228:8000/tcmid/) [32]. The component structures obtained from the PubChem (https://pubchem.ncbi.nlm.nih.gov/) [33] and TCMSP databases were input into the SwissTargetPrediction database (http://www.swisstargetprediction.ch/) [34] for the prediction of the underlying target genes of main components in Xiaoji recipe.

### 2.7. Exploration of Potential Targets of Pancreatic Cancer

The potential target genes of pancreatic cancer were searched in the Disgenet (https://www.disgenet.org/) [35], OMIM (https://omim.org/) [36], and Genecards (https://www.genecards.org/) [37] databases using the “pancreatic ductal adenocarcinoma” as the keyword.

### 2.8. The Screening of Component-Disease Targets and Network Construction

The 522 targets of Xiaoji recipe and 998 targets of pancreatic cancer were imported into the Venny2.1 software, and the obtained Venn diagram showed 116 shared targets of the pancreatic cancer and the components of Xiaoji recipe. The drug-component-target-disease network was constructed using the Cytoscape 3.8.2 software and analyzed with the Network Analyzer function. The hub genes were analyzed and selected based on the topological analysis, and the degree value indicates the relation between the components and targets (Table 1).

### 2.9. Protein–Protein Interaction (PPI) Network Construction

The interaction of the 116 component-disease targets was explored on the STRING platform (https://cn.string-db.org/) [38] under “*Homo sapiens*.” The protein was presented as nodes, and the association between proteins was shown as edges in the PPI network, and the size and shade of color represented the value of degree. Furthermore, based on the topological analysis, the results from the STRING database were analyzed with the Cytoscape 3.8.2 software using the Network Analyzer function, and the core targets were selected under the condition of degree value over the average. The top 30 targets were selected and exported the bar graph using the R 4.0.5 software. Based on the clustering analysis, the results from the STRING database were imported into the Cytoscape 3.8.2 software and analyzed using the Molecular Complex Detection (MCODE) plugin. Three gene clusters were obtained, and 2 core genes (HSP90AA1, CDK6) were selected.

### 2.10. GO and KEGG Functional Enrichment Analysis

Gene Ontology (GO) analysis including the biological process (BP), molecular function (MF), and cellular components (CC) and the biological pathway (KEGG) enrichment analysis of 116 disease-component targets were performed using the R software with Bioconductor package under *p* value < 0.05. The results were exported with the bar graphs and pathway maps.

### 2.11. Statistical Analysis

All experiments were completed three times independently. The results were analyzed using GraphPad 8 software and presented as the mean ± SD. Student's *t*-test was used to compare the difference between two groups, and one-way ANOVA was used for multiple group comparisons. *p* < 0.05 indicates statistical significance.

## 3. Results

### 3.1. Active Ingredients and Their Potential Targets in Xiaoji Recipe

We found 32 potential active ingredients of Xiaoji recipe *Curcuma zedoaria* (E Zhu), *Polygonum cuspidatum* (Huzhang), *clematis root* (Weilingxian), *Rhizoma Paridis* (Zhonglou) and *Eupolyphaga Steleophaga* (Tubiechong) based on the TCMSP database, under OB ≥ 30% and DL ≥ 0.18 and TCMID database (Table 2). There were 3 ingredients from *Curcuma zedoaria*, 10 ingredients from *Polygonum cuspidatum*, 7 ingredients from *clematis root*, 10 ingredients from *Rhizoma Paridis*, and 4 ingredients from *Eupolyphaga Steleophaga* (Table 3). *Curcuma zedoaria*, *Polygonum cuspidatum*, and *clematis root* share the same ingredient beta-sitosterol. Based on the SwissTargetPrediction platform, we performed the prediction of the potential targets of active components in *Curcuma zedoaria* (E Zhu), *Polygonum cuspidatum* (Huzhang), *clematis root* (Weilingxian), *Rhizoma Paridis* (Zhonglou), and *Eupolyphaga Steleophaga*. Totally, 522 target genes of these active ingredients of Xiaoji recipe were screened out, and there were 159 targets for *Curcuma zedoaria*, 313 targets for *Polygonum cuspidatum*, 107 targets for *clematis root*, 271 targets for *Rhizoma Paridis*, and 44 targets for *Eupolyphaga Steleophaga* (Table 3).

### 3.2. Construction of the Target Gene Network of Pancreatic Cancer and Xiaoji Recipe

We searched the potential targets in the OMIM, Disgenet, and Genecards using the keywords “pancreatic ductal adenocarcinoma,” and totally, 998 potential targets of PDAC were obtained. Venny 2.1 software was used to select the shared targets for PDAC and Xiaoji recipe, and the results showed that there were 116 shared targets in the intersection area (Figure 1(a)). Then, the 32 active ingredients in Xiaoji recipe and 116 compound-disease targets were input into the Cytoscape 3.8.2 software, and we deleted 4 isolated components that were not intersected with the targets. The remaining 28 active components were marked in red in Table 2. The main active biomolecules were analyzed using the Network Analyzer function. As shown in Figure 1(b), the red button represented the disease, the blue bubbles represented the 116 compound-disease targets, the purple rectangle represented the Chinese medical materials, and the green triangles represented the 28 active ingredients in Xiaoji recipe. The top five core ingredients were bisdemethoxycurcumin, luteolin, quercetin, flavone, and beta-ecdysone, as shown in Table 1.

### 3.3. Construction of the PPI Network and Analysis of Targets

The PPI network was constructed based on the STRING database and Cytoscape software to investigate the underlying interaction among the 116 targets. Based on the topology analysis, the 116 compound-disease targets were input in the STRING platform for the protein-protein interaction network construction. There were 116 nodes and 2210 edges (Figure 2(a)). Further, the interaction data from the STRING database were imported into the Cytoscape software for the interaction network. The degree was determined by the size and color shade of the nodes (Figure 2(b)). TP53, HRAS, VEGFA, AKT1, STAT3, EGFR, and SRC were the core target genes.

The hub genes in the network were identified by the top 30 targets ranked by degree on the PPI network, which was performed using the R 4.0.5 software as shown in Figure 3(a). Moreover, based on the clustering analysis and analysis using Cytoscape software, three gene clusters were obtained with two core target genes, HSP90AA1 and CDK6, which were potentially involved in the development of PDAC (Figure 3(b)).

### 3.4. GO and KEGG Pathway Enrichment Analysis

Based on the GO enrichment analysis, the biological process, cellular component, and molecular function of the 116 component-disease targets were analyzed using R software. The results revealed that the target genes were enriched in 2144 BP, 50 CC expression process, and 132 MF-related process. The biological functions of targets mainly included the peptidyl-serine modification and phosphorylation, positive modulation of protein serine/threonine kinase activity and MAP kinase activity, and gland development (Figure 4). The molecular functions mainly included the protein tyrosine kinase activity, phosphatase binding, insulin receptor substrate binding, and growth factor binding (Figure 5). The cellular component mainly included the transferase complex, protein kinase complex, serine/threonine protein kinase complex, membrane raft, and transcription regulator complex (Figure 6).

A total of 159 KEGG signaling pathways of the 116 shared target genes were obtained using the R software. The top 20 significant signaling pathways were shown in histograms. The results revealed that these targets were closely associated with the PI3K-AKT pathway, EGFR tyrosine kinase inhibitor resistance, endocrine resistance and MAPK signaling, and pancreatic cancer, which may improve the understanding of the molecular mechanism associated with pancreatic cancer progression (Figure 7). Moreover, the target genes involved in the PI3K-AKT and MAPK signalings in pancreatic cancer were shown in Figures 8(a) and 8(b).

### 3.5. Xiaoji Recipe Inhibited the Proliferation and Migration of Pancreatic Cancer Cells

Furthermore, we explored the effects of Xiaoji recipe on the malignant behaviors of pancreatic cancer cells. As revealed by the CCK-8 assay, the viability of CFPAC and PANC1 cells exhibited significant reduction with Xiaoji recipe treatment in a concentration-dependent way (Figures 9(a) and 9(b)). Furthermore, we conducted wound healing assays to explore the impact of Xiaoji recipe on pancreatic cancer cell migration. The results demonstrated that the migration ability of CFPAC and PANC1 was significantly suppressed by the treatment of Xiaoji recipe, and the higher the concentration, the more significant the suppression (Figures 9(c) and 9(d)).

### 3.6. Xiaoji Recipe Promoted the Apoptosis of Pancreatic Cancer Cells In Vitro

The effects of Xiaoji recipe on the apoptosis of pancreatic cancer cells were explored using flow cytometry analysis. As shown in Figures 10(a) and 10(b), the apoptosis rate of CFPAC and PANC1 cells were continuously elevated as the concentration of Xiaoji recipe increased, which indicated that Xiaoji recipe facilitated pancreatic cancer cell apoptosis in a dose-dependent way.

### 3.7. Xiaoji Recipe Exerted Inhibitory Effects on the Activation of AKT, MAPK, and STAT3 Signaling Pathways

Whether Xiaoji recipe affected the activation of AKT, MAPK, and STAT3 signaling pathways was further explored. The protein expression of AKT1, STAT3, EGFR, and MAPK3 in pancreatic cancer cells was detected using Western blot. We found that the AKT1, STAT3, EGFR, and MAPK3 protein expression showed significant decrease in CFPAC and PANC1 cells after Xiaoji recipe treatment in a dose-dependent manner (Figures 11(a) and 11(b)).

## 4. Discussion

Pancreatic cancer, as one of the most fatal malignancies, is reported with increasing incidence in recent years. The prognosis of pancreatic cancer patients is still unsatisfying due to the atypical early symptoms and distal metastasis [39]. Thus, it is imperative to explore the underlying mechanism of pancreatic cancer pathogenesis. In our work, the primary active components of Xiaoji recipe and the potential targets and mechanisms in the treatment of pancreatic cancer were investigated based on network pharmacology. The exploration of underlying mechanism of Xiaoji recipe may provide evidence for the TCM therapy in pancreatic cancer.

Chinese herbal medicine (CHM) is indicated as a promising treatment option for multiple malignant diseases with unique clinical effects [40, 41]. As reported previously, Xiaoji recipe has been to inhibit cell migration and growth of lung adenocarcinoma and gastric cancer [42, 43]. Consistently, our study found that Xiaoji recipe repressed cell proliferation and migration while promoted cell apoptosis in pancreatic cancer. More importantly, the main active components of Xiaoji recipe were explored in our study. Bisdemethoxycurcumin, luteolin, quercetin, flavone, and beta-ecdysone were the top five active ingredients ranked by degree according to the component-target-disease network, which were potentially the main active ingredients in the treatment of pancreatic cancer. Bisdemethoxycurcumin is reported with antifibrosis, antiapoptosis, antioxidant, and anti-inflammatory characteristic in various diseases [44–46]. Bisdemethoxycurcumin is also reported with antitumor effects in hepatocellular carcinoma, breast cancer, and non-small-cell lung cancer [47–49]. Luteolin is a flavonoid with anti-inflammation, antiallergy, and anticancer properties and suppresses cell transformation, metastasis, invasion, and angiogenesis in carcinogenesis [50–52]. It has also been reported to inhibit the invasion and epithelial-mesenchymal transition of pancreatic cancer cells by inactivating the STAT3 pathway [53]. Quercetin is reported with cytotoxic and antitumor effects and suppresses pancreatic cancer progression by inhibiting the STAT3 pathway activation [54]. The active ingredients possess different degrees of therapeutic effects on pancreatic cancer and are involved in various signaling pathways.

The component-disease network showed the target genes regulated by these active components in pancreatic cancer. The genes include EGFR, CDK1, MMP7, BCL2, and PARP1. Moreover, the PPI networks revealed that TP53, HRAS, VEGFA, AKT1, STAT3, EGFR, and SRC were the core target genes in the PPI network. The target genes were not mutually independent but were interacted with each other. The Xiaoji recipe may inhibit the progression of pancreatic cancer by regulating the multiple proteins. In line with our finding, all mentioned core target genes have been reported as major driver genes for pancreatic cancer [55–60].

GO and KEGG enrichment analysis revealed the biological process, molecular functions, cellular component as well as the related signaling pathways in the occurrence and progression of pancreatic cancer. There were 2144 BP, 50 CC expression process, and 132 MF-related process of these 116 component-disease targets. We also found that the enrichment of the 116 component-disease targets in the PI3K/AKT and MAPK pathways according to the KEGG analysis. PI3K/AKT pathway is critically involved in the regulation of malignant behaviors in pancreatic cancer, indicating that PI3K/AKT is a valuable target for pancreatic cancer therapy [30, 61]. The MAPK pathways are reported to regulate the tumor cell proliferation, differentiation, apoptosis, and resistance to drug therapy, and PI3K/AKT and Ras/MEK/MAPK pathways were the two main signaling in the downstream of EGFR [62]. In our study, we found that EFGR is one of the component-disease targets, and Xiaoji recipe may inhibit the activation of MAPK signaling by targeting EFGR in pancreatic cancer. In addition, we performed in vitro assays to demonstrate that Xiaoji recipe exerted inhibitory effects on the activation of PI3K/AKT, MAPK, and STAT3 signaling pathways. For all we know, these three signaling pathways are widely reported in the involvement of pancreatic cancer. Moreover, many literatures have supported that TCMs inhibit tumor progression via these signaling pathways [63–65].

In this study, the active ingredients and related targets of Xiaoji recipe in pancreatic cancer were explored, and the biological process, molecular function, cellular process, and related signaling pathways were under investigation based on the network pharmacology approach. Moreover, we also verified the effect of Xiaoji recipe on pancreatic cancer cell proliferation, migration, apoptosis, and relevant signaling pathways using in vitro assays. Xiaoji recipe significantly inhibited the proliferation, migration, AKT, MAPK, and STAT3 signaling pathways and induced the apoptosis of pancreatic cancer cells, which indicated its potential in clinical therapy of pancreatic cancer patients.

However, our study also exists some limitations. First, the in vivo experiments of Xiaoji recipe on tumor growth were lack. Second, the specific mechanism of Xiaoji recipe on regulating the PI3K/AKT, MAPK, and STAT3 signaling pathways were not explored. More, the potential mechanism of Xiaoji recipe on regulating the core target genes of TP53, HRAS, VEGFA, AKT1, STAT3, EGFR, and SRC in pancreatic cancer were not shown. All these limitations will be perfected in the near future.

## Figures and Tables

**Figure 1:** Construction of the target gene network of pancreatic cancer and Xiaoji recipe. (a) The Venn diagram of potential targets of main active components in Xiaoji recipe and pancreatic cancer. (b) The component-disease target network.

**Figure 2:** Construction of the PPI network and analysis of targets of Xiaoji recipe in pancreatic cancer. (a) The PPI network of 116 compound-disease target genes. (b) The topological analysis of the 116 compound-disease target genes.

**Figure 3:** The analysis of compound-disease hub genes. (a) The top 30 genes from the PPI network based on the topological analysis. (b) The clustering analysis of the PPI network.

**Figure 4:** GO analysis for biological process of component-disease targets.

**Figure 5:** GO analysis for molecular function of component-disease targets.

**Figure 6:** GO analysis for cellular component of component-disease targets.

**Figure 7:** KEGG enrichment analysis of the Xiaoji recipe potential targets in pancreatic cancer.

**Figure 8:** The related signaling pathways of component-disease targets. (a) The potential targets in MAPK signaling pathway. (b) The potential targets in PI3K/AKT signaling pathway.

**Figure 9:** The effect of Xiaoji recipe on cell viability and migration in pancreatic cancer. (a) CCK-8 assays were used to evaluate the viability of CFPAC and PANC1 cells after the treatment of different concentrations of Xiaoji recipe. (b) The migration of CFPAC and PANC1 cells after indicated treatments was subject to wound healing assays. ^∗∗^*p* < 0.01.

**Figure 10:** The effect of Xiaoji recipe on pancreatic cancer cell apoptosis. (a) The apoptosis rate of CFPAC and PANC1 cells after indicated treatments was subject to flow cytometry analysis.

**Figure 11:** The effect of Xiaoji recipe on MAPK and PI3K/AKT signaling pathways. (a, b) The protein expression of AKT, STAT3, EGFR, and MAPK3 in CFPAC and PANC1 cells after indicated treatments.

**Table 1:** Relation between potential targets and active components in Xiaoji recipe.

Component name	Degree	Betweenness centrality	Closeness centrality	Eccentricity
Bisdemethoxycurcumin	36	0.049102808	0.422096317	4
Luteolin	31	0.024267623	0.408219178	4
Quercetin	30	0.021502194	0.403794038	4
Flavone	30	0.029632826	0.412742382	4
Beta-ecdysone	27	0.02982601	0.40599455	4
Physovenine	22	0.016298752	0.38501292	4
(4aS,6aR,6aS,6bR,8aR,10R,12aR,14bS)-10-hydroxy-2,2,6a,6b,9,9,12a-heptamethyl-1,3,4,5,6,6a,7,8,8a,10,11,12,13,14b-tetradecahydropicene-4a-carboxylic acid	18	0.011697317	0.37913486	4
Pennogenin	18	0.008901981	0.375314861	5
ClematosideA′_qt	17	0.010539948	0.37721519	4
Picralinal	16	0.007242384	0.373433584	4
Rhein	16	0.009358031	0.371571072	4
Pennogenin VI	16	0.006015765	0.371571072	5
Pennogenin VII	16	0.006015765	0.371571072	5
6,8-Dihydroxy-7-methoxyxanthone	14	0.005718922	0.362530414	4
Physciondiglucoside	11	0.005127525	0.362530414	4
Diosgenin	10	0.002912114	0.357314149	5
Beta-sitosterol	9	0.011919371	0.355608592	4
Polysaccharide	9	0.003448702	0.347319347	5
Hederagenin	8	0.004162798	0.357314149	4
Stigmasterol	6	0.00185844	0.347319347	4
Wenjine	5	0.001187609	0.326039387	5
Cholesterol	5	0.005333285	0.344110855	4
Embinin	4	0.001738369	0.337868481	5
Dioscin I	4	3.06*E*-04	0.333333333	5
Dioscin II	4	3.06*E*-04	0.333333333	5
Torachrysone-8-O-beta-D-(6′-oxayl)-glucoside	3	2.64*E*-04	0.334831461	5
Heptyl phthalate	3	7.37*E*-04	0.336343115	4
Pariphyllin	3	1.43*E*-04	0.328918322	5

**Table 2:** Active ingredients of Xiaoji recipe.

Mol ID	Molecule name	OB (%)	DL	Chinese medicinal materials
MOL000296	Hederagenin	36.91	0.75	*Curcuma zedoaria*
MOL000906	Wenjine	47.93	0.27	*Curcuma zedoaria*
MOL000940	Bisdemethoxycurcumin	77.38	0.26	*Curcuma zedoaria*
MOL013281	6,8-Dihydroxy-7-methoxyxanthone	35.83	0.21	*Polygonum cuspidatum*
MOL013287	Physovenine	106.21	0.19	*Polygonum cuspidatum*
MOL013288	Picralinal	58.01	0.75	*Polygonum cuspidatum*
MOL002259	Physciondiglucoside	41.65	0.63	*Polygonum cuspidatum*
MOL002268	Rhein	47.07	0.28	*Polygonum cuspidatum*
MOL002280	Torachrysone-8-O-beta-D-(6′-oxayl)-glucoside	43.02	0.74	*Polygonum cuspidatum*
MOL000358	Beta-sitosterol	36.91	0.75	*Polygonum cuspidatum*, *clematis root*, *Eupolyphaga Steleophaga*
MOL000492	(+)-catechin	54.83	0.24	*Polygonum cuspidatum*
MOL000006	Luteolin	36.16	0.25	*Polygonum cuspidatum*
MOL000098	Quercetin	46.43	0.28	*Polygonum cuspidatum*
MOL001663	(4aS,6aR,6aS,6bR,8aR,10R,12aR,14bS)-10-hydroxy-2,2,6a,6b,9,9,12a-heptamethyl-1,3,4,5,6,6a,7,8,8a,10,11,12,13,14b-tetradecahydropicene-4a-carboxylic acid	32.03	0.76	*Clematis root*
MOL002372	(6Z,10E,14E,18E)-2,6,10,15,19,23-hexamethyltetracosa-2,6,10,14,18,22-hexaene	33.55	0.42	*Clematis root*
MOL000449	Stigmasterol	43.83	0.76	*Clematis root*
MOL005594	ClematosideA′_qt	37.51	0.76	*Clematis root*
MOL005598	Embinin	33.91	0.73	*Clematis root*
MOL005603	Heptyl phthalate	42.26	0.31	*Clematis root*
	Dioscin I			*Rhizoma Paridis*
	Dioscin II			*Rhizoma Paridis*
	Diosgenin			*Rhizoma Paridis*
	Flavone			*Rhizoma Paridis*
	Pariphyllin			*Rhizoma Paridis*
	Pennogenin			*Rhizoma Paridis*
	Pennogenin VI			*Rhizoma Paridis*
	Pennogenin VII			*Rhizoma Paridis*
	Polysaccharide			*Rhizoma Paridis*
	Beta-ecdysone			*Rhizoma Paridis*
	Cholesterol			*Eupolyphaga Steleophaga*
	Flavacin			*Eupolyphaga Steleophaga*
	Hypoxanthine			*Eupolyphaga Steleophaga*

**Table 3:** Active ingredients and their potential targets in Xiaoji recipe.

Name	Ingredients (*n*)	Predicted targets (*n*)
*Curcuma zedoaria* (Ezhu)	3	159
*Polygonum cuspidatum* (Huzhang)	10	313
*Clematis root* (Weilingxian)	7	107
*Rhizoma Paridis* (Zhonglou)	10	271
*Eupolyphaga Steleophaga* (Tubiechong)	4	44

## Data Availability

Data generated in this study are available from the corresponding author under reasonable requests.
